# SCU-Net: Semantic Segmentation Network for Learning Channel Information on Remote Sensing Images

**DOI:** 10.1155/2022/8469415

**Published:** 2022-04-10

**Authors:** Wei Wang, Yuxi Kang, Guanqun Liu, Xin Wang

**Affiliations:** ^1^School of Computer and Communication Engineering, Changsha University of Science and Technology, Changsha 410114, China; ^2^Hunan Open University, Changsha 410004, China

## Abstract

Extracting detailed information from remote sensing images is an important direction in semantic segmentation. Not only the amounts of parameters and calculations of the network model in the learning process but also the prediction effect after learning must be considered. This paper designs a new module, the upsampling convolution-deconvolution module (CDeConv). On the basis of CDeConv, a convolutional neural network (CNN) with a channel attention mechanism for semantic segmentation is proposed as a channel upsampling network (SCU-Net). SCU-Net has been verified by experiments. The mean intersection-over-union (MIOU) of the SCU-Net-102-A model reaches 55.84%, the pixel accuracy is 91.53%, and the frequency weighted intersection-over-union (FWIU) is 85.83%. Compared with some of the state-of-the-art methods, SCU-Net can learn more detailed information in the channel and has better generalization capabilities.

## 1. Introduction

Remote sensing image processing technology has developed rapidly. The image semantic segmentation approach based on CNN has become a hot research direction in satellite remote sensing image semantic segmentation [1], and it is widely used in land detection, vegetation classification, environmental monitoring, urban planning, national defense security, and other fields. At the same time, the neural network can automatically obtain the information contained in the pictures and accurately predict the category of unknown data [2]. Therefore, academia began to use neural networks to obtain the deep features in high-resolution remote sensing images and use them for satellite remote sensing image classification [3].

Recently, the deep learning method has performed well in the computer vision recognition task, and CNN has achieved very good results in image classification [4–9], semantic segmentation [10], and target detection [11, 12]. The realization of LeNet [13] established the structure of CNN, and classic CNNs, such as VGG [14], GoogleNet [15], and ResNet [16] have made great achievements. FC-DenseNet (fully convolutional DenseNet) was proposed by Simon et al. [17] to enhance feature extraction and feature reuse. Based on a fully convolutional network, the standard convolutional layer is replaced by dense block [18], and the resulting network can achieve new pixel-level segmentation tasks rather than traditional image classification tasks. To make the output size of the network equal to the input size, the upsampling structure of FCN is added. The network achieves a good segmentation effect in semantic segmentation. The DFCN (dense fully convolutional network) proposed by Wang et al. [19], which also combined DenseNet and fully convolutional network, introduced the dense blocks in the dense network into the full convolutional network. Finally, a good segmentation effect has been achieved on the satellite remote sensing image dataset.

There are many important methods of image processing, among which image semantic segmentation is one. Semantic segmentation is to divide the pixels in the image and predict the category of each pixel in the image using the neural network [20], which is like image super-resolution reconstruction [21]. Recently, geographic information system (GIS), self-driving car, medical image analysis, and robot have become the main application fields of semantic segmentation. This paper mainly studies the application of semantic segmentation methods in the field of geographic information systems. There have been many pieces of research on semantic segmentation using deep learning methods in recent years. The development and application of CNN [5] are introduced by Long et al. In 2015, the FCN for image semantic segmentation was proposed by Long [10]. It adjusts the structure of the ordinary convolution network and realizes the intensive prediction of the image by abandoning the fully connected layer. At the same time, a skip connection is added to the network. This method can not only extract the rough semantic information from the deep layer but also combine the appearance information from the shallow layer, which makes the segmentation more refined. The FCN convolution neural network is used to realize the leap from image pixels to pixel categories. For the medical image segmentation problem, inspired by the FCN network, Fischer et al. proposed U-Net [22]. Through the design of a U-shaped network structure in U-net, not only context information but also location information can be obtained, which has achieved good results in biomedical segmentation applications. U-Net won the first prize for outstanding performance in the 2015 ISBI cell tracking competition. SegNet [23] was proposed by Badrinarayanan et al. It is based on the encoder-decoder structure, which reduces the number of network parameters by discarding the location information in the pooling layer during the upsampling process and achieves good results. The researchers conducted experiments on two datasets, one is the SUN RGB-D dataset used for indoor scene segmentation. The other is the use of the CamVid dataset for road scene segmentation. The DeepLab series network was proposed by Google. DeepLabV1 [24] is an improved semantic segmentation network based on VGG16. Researchers found in experiments that the accuracy of using deep convolutional neural networks in the field of semantic segmentation is insufficient. The translation invariance of the advanced features of deep convolutional neural networks is the fundamental reason. DeepLabv1 combines a fully connected conditional random field (CRF) with the response of a deep convolutional neural network to try to solve this problem. Then, the Hole (dilated convolution) algorithm is creatively integrated into the deep convolution neural network model, which performs well on the PASCAL VOC 2012 dataset. An image segmentation algorithm based on spatial pyramid pool (ASPP) structure was proposed by DeepLabV2 [25]. ASPP can capture the contextual content of objects and images at multiple scales and detect incoming convolution features using convolution kernels with multiple sampling rates and effective field of view. DeepLabv2 further highlights the role of hole convolution in dense prediction tasks. In the deep convolution network, the dilated convolution can effectively control the resolution (receptive field) of calculating the feature responses to effectively expand the receptive field of convolution kernels without additional parameters or calculation. Integrate more context information. DeepLabV3 [26] uses the multigrid strategy and adds batch normalization, global pooling layer, point convolution layer, and bilinear interpolation upsampling to the ASPP module, achieving good results. The DeepLabV3+ [27] network uses the Xception [28] network as the backbone and uses the encoder-decoder structure. In addition, both [29, 30] use support vector machine (SVM) to segment remote sensing images.

Inspired by these studies, this paper proposes a new method for semantic segmentation of satellite remote sensing images. In the task of semantic segmentation of satellite remote sensing images, the improved upsampling method proposed in this paper not only reduces the number of model parameters but also improves the recognition ability of the model. Based on the new upsampling module, a novel image semantic segmentation model and introduced attention mechanism are proposed. In addition, a new remote sensing image dataset is provided, which shows the remote sensing information of Chenzhou, China. These satellite remote sensing images come from China's GF-2 satellite with a spatial resolution of 0.8 meters, showing various spatial information of cultivated land, forest land, waters, buildings, etc. The original images in the dataset are labeled based on local geomorphological features. Finally, the method in this article was tested on this dataset. Compared with other semantic segmentation methods based on deep learning, SCU-Net has better segmentation performance and stronger generalization ability.

## 2. SCU-Net

This section will, firstly, introduce the structure of FCN. Secondly, the structure and principle of SCU-Net proposed in this paper are introduced. Finally, the network complexity of SCU-Net is analyzed through experiments.

### 2.1. Fully Convolutional Network

The main difference between the FCN network and the traditional deep learning convolutional network is that it does not use a full connection layer. The FCN network adds an upsampling method to the network structure. The output image has the same size as the original input image, which realizes pixel classification. FCN is mainly composed of the feature extraction module of the ordinary convolutional network, upsampling, and skip connection.  Figure 1 shows the structure of FCN, where “Input” represents the input end of the image, and “Conv1,” “Conv2,” “Conv3,” “Conv4,” and “Conv5” represent ordinary convolutional layers. “MaxPooling” means the pooling layer. “Upsampling-1” means 2 times the upsampling module, “Upsampling-2” means 4 times the upsampling module, “Upsampling-3” means 8 times the upsampling module, and three upsampling modules can process the feature map to 2 times, 4 times, and 8 times the size of the original image.

The first operation is feature extraction. If the input image size is *H* × *W*, the original image will be reduced to (*H* × *W*)/2 after the “Conv1” and “MaxPooling” operations. Then, the feature map is reduced to (*H* × *W*)/4 through the operations of “conv2” and “MaxPooling.” By using the “Conv3” and “MaxPooling” operations, the output feature map “featureMap-3” with reduced size (*H* × *W*)/8 can be obtained. Then, “Conv4” and “MaxPooling” operations are performed to reduce the size of the feature map to (*H* × *W*)/16, and the output feature map is named “featureMap-4.” In the next step, the feature map goes through “Conv5” and the last “MaxPooling” operation, and the feature map, namely “featureMap-5,” will be reduced to (*H* × *W*)/32.

After the feature extraction is completed, the upsampling operation is performed. First, the “Upsampling-1” operation is performed on “featureMap-4” to obtain a feature map “featureMap-6” with a size of (*H* × *W*)/8. Next, “featureMap-5” performs the “Upsampling-2” operation to obtain the feature map “featureMap-7” whose size is (*H* × *W*)/8. Then, “featureMap-6” and “featureMap-7” are stitched together. Finally, the “Upsampling-3” operation is performed on the output result to output the feature map. The size of this feature map is the same as the original image, and the semantic segmentation is completed.

### 2.2. Network Structure

The channel feature weight extraction module (CFWE) [7]is introduced to improve the feature extraction ability of the semantic segmentation network model.  Figure 2 is the detailed structure of CFWE. In this structural diagram, “Convk” denotes a convolutional layer with a filter size of *k*, where *k* is equal to 3 or 1. “GAP” denotes the global average pooling layer, and “FC” denotes the full connected layer.

The CFWE module is a multilayer structure. The first is the short connections layer of the CFWE. It contains 3 convolutional layers, of which, there are two conv1 and one conv3. The two “conv1” in the module are used to increase and decrease the number of channels, respectively, with the purpose of reducing the amounts of parameters. The shortcut connections layer can alleviate the network degradation problem to a certain extent. Next comes the serial pool layer and full connection layer structure, which consists of two “FC” structures and a “GAP” structure. Firstly, the feature map of each channel is processed as a global feature using the “GAP” structure. Then, the feature dimension is reduced through the first “FC” layer, and the feature dimension is restored by the second “FC” layer. The weight coefficient model of each channel can be learned after passing through two “FC” layers. Finally, the final output feature map is to multiply the original feature and the extracted feature map channel weight coefficients by short connections. When extracting features, the weight coefficient is useful for the model to extract more important channel features and then enhance the feature extraction ability of the network.

In the traditional semantic segmentation neural network, the upsampling step is divided into two steps. Firstly, the feature map size is up-sampled to the original image size, and then point convolution is performed to complete the semantic segmentation. The parameters and calculations of the network model using this method are relatively large. The “CDeConv” module proposed, firstly, performs point convolution to make the number of feature map channels consistent with the number of segmentation task categories, and then, it performs deconvolution to make the output feature map size consistent with the original image size. This module not only reduces the number of model calculations and parameters but also improves model performance. Its structure is shown in Figure 3.

According to the CFWE module and the “CDeConv” module, a novel semantic segmentation network model SCU-Net is proposed, whose structure is shown in Figure 4. Among them, “Input” represents the input image, and “Output” represents the output result. “Conv” not only includes “Convolution,” but also “Batch Normalization” and “Activation Function.” The function of this composite structure is to extract image features. “Conv7” is a “Conv” structure with *k* equal to 7 and a stride equal to 2. “Conv1” is a “Conv” structure with *k* equal to 1 and a stride equal to 1. “Conv1-3-1” is a structure consisting of “Conv1,” “Conv3,” and “Conv1” in series. One of the two “Conv1” structures is used to increase the dimensionality and the other can decrease the dimensionality. This operation can reduce the complexity of the model. “Conv3” is used for feature extraction. “Maxpooling” means the maximum pooling layer with a step size of 2 and a window size of 3. Its main function is to upsample, reduce dimensionality, and reduce the amount of calculation. “Upsampling” represents an 8 times upsampling module, and its function is to upsample the feature map to the same size as the original image to achieve semantic segmentation.

If the input image is *X* and the size is *H* × *W* × 3, it, firstly, passes through the “Conv7” module with 64 convolution kernels. The step size is 2, and the convolution kernel size is 7. Set the output feature map of the “Conv7” module to *X*1. The size becomes *H*/2 × *W*/2 × 64, which is shown as follows:

(1) $$\begin{array}{c} X1=\mathrm{Conv}7\left(X\right). \end{array}$$

After a maxpool layer, the number of channels will not change, however, the size of the output feature map *X*2 will become 0.25 times that of *X*1, as shown below.

(2) $$\begin{array}{c} X2=\mathrm{MaxPooling}\left(X1\right). \end{array}$$

Then, through *n* (*n* is a settable parameter, related to the number of network layers) serially connected “Conv1_3_1,” the output size of the feature map is *H*/4 × *W*/4 × 256. Next, the output *X*_3_ can be obtained by using CFWE module. Its feature map size is *H*/4 × *W*/4 × 256, which can be expressed as follows:

(3) $$\begin{array}{c} X3=\mathrm{CWFE}\left(\mathrm{Conv}1\_3\_1\left(\mathrm{Conv}1\_3\_1\left(......\left(X2\right)\right)\right)\right). \end{array}$$

After that, the feature map *X*3 is input to the *n* series of “Conv1_3_1” modules, and then through a layer of CFWE module, the output feature map *X*4 has a size of *H*/8 × *W*/8 × 512, which can be expressed as follows:

(4) $$\begin{array}{c} X4=\mathrm{CWFE}\left(\mathrm{Conv}1\_3\_1\left(\mathrm{Conv}1\_3\_1\left(......\left(X3\right)\right)\right)\right). \end{array}$$

The feature map *X*4 is input to the *n* series of “Conv1_3_1” modules, and then through a layer of CFWE module, the output feature map *X*5 size is *H*/16 × *W*/16 × 1024, which can be expressed as follows:

(5) $$\begin{array}{c} X5=\mathrm{CWFE}\left(\mathrm{Conv}1\_3\_1\left(\mathrm{Conv}1\_3\_1\left(......\left(X4\right)\right)\right)\right). \end{array}$$

Then, the feature map *X*5 is input to *n* serially connected “Conv1_3_1” modules, and the output feature map *X*6 has a size of *H*/32 × *W*/32 × 2048, which can be expressed as follows:

(6) $$\begin{array}{c} X6=\mathrm{CWFE}\left(\mathrm{Conv}1\_3\_1\left(\mathrm{Conv}1\_3\_1\left(......\left(X5\right)\right)\right)\right). \end{array}$$

The feature map *X*6 uses a CDeConv module to perform point convolution, firstly, to achieve the purpose of reducing the number of channels, reducing the number of channels to 7. Then, upsample 4 times, and get the output *X*7. Its feature map size is *H*/8 × *W*/8×7, which can be expressed as follows:

(7) $$\begin{array}{c} X7=\mathrm{CDeConv}\left(X6\right). \end{array}$$

Feature map *X*5 enters a CDeConv module through a skip connection. Firstly, point convolution is performed to reduce the number of channels to 7. Then, upsample 2 times. Get the output *X*7′. Its feature map size is *H*/8 × *W*/8 × 7, which can be represented as follows:

(8) $$\begin{array}{c} X7{}^{\prime }=\mathrm{CDeConv}\left(X5\right). \end{array}$$

The feature map *X*4 reduces the number of channels to 7 through a point convolution, and the size of the output feature map *X*7″ is *H*/8 × *W*/8 × 7, which can be represented as follows:

(9) $$\begin{array}{c} X7{}^{\prime \prime }=\mathrm{CDeConv}\left(X4\right). \end{array}$$

Then, add *X*7, *X*7′, and *X*7″ bit-by-bit to get *X*8. Its feature map size is *H*/8 × *W*/8 × 7, which can be expressed as follows:

(10) $$\begin{array}{c} X8=X7⊕X7{}^{\prime }⊕X7{}^{\prime \prime }. \end{array}$$

The final feature map *X*_8_ passes an 8 times upsampling module to output the final output feature map, whose size is *H* × *W* × 7, and can be expressed as

Three different upsampling methods using different numbers of “CDeConv” modules and skip connections are designed. Figure 4 shows SCU-Net-A. Based on SCU-Net-A, the network obtained by deleting the first “Conv1” module and a corresponding skip connection on the network backbone is SCU-Net-B. Based on SCU-Net-B, the network obtained by removing a “CDeConv” module connected to the CFWE module is SCU-Net-C.

Based on SCU-Net, combined with data expansion technology for image preprocessing, an automatic remote sensing image segmentation method is proposed.  Figure 5 shows the specific process of the network model. Firstly, preprocess the remote sensing image data, and then it is input into SCU-Net for image semantic segmentation, and finally, the network outputs the segmented image.

### 2.3. Network Complexity

Model complexity refers to the amount of calculation and parameters of the network. The parameters and calculations of different upsampling methods and depth models are compared through the experiments. Experiments were performed with one “CDeConv,” two “CDeConv,” and three “CDeConv” modules in the network model using three different upsampling methods. By combining three different upsampling methods and three different network depths, we can get 9 different network models.  Figure 6 is a comparison diagram of parameter quantities.  Figure 7 is a comparison chart of the number of calculations.

As shown in Figure 6, when the depth of the SCU-Net is the same, the parameters of the C structure are about 10,000 less than the network parameters of the A and B structures. It shows that different upsampling structures have little influence on the parameters of the network model. The parameter quantity of SCU-Net-153-A is 2.46 times that of SCU-Net-51-A, and the parameter quantity of SCU-Net-102-A is 1.80 times that of SCU-Net-51-A. Therefore, it can be inferred that the number of model parameters is most affected by the number of network layers. Therefore, when the equipment does not support a large parameter scale, it is better to use a shallow depth network model.

The floating point of operations refers to the number of multiplication and addition operations in the model. As shown in Figure 7, the depth of the network has a great influence on the amount of calculation. As far as the amount of calculation is concerned, SCU-Net-153 is 1.44 times that of SCU-Net-102, and SCU-Net-102 is 1.78 times that of SCU-Net-51. The calculation amount of SCU-Net-153 and SCU-Net-102 is very huge. Therefore, when the model accuracy gap is small, the SCU-Net-51 model has the lowest cost.

## 3. Experimental Results

### 3.1. Dataset

This experimental dataset comes from the fusion image of GF-2 in the Chenzhou area in 2016. As shown in Figure 8, there are satellite remote sensing images in the dataset. The landform of the Chenzhou area is complex, and the forest is rich in plant species. The number of wavebands is 3, and the spatial resolution of this remote sensing image is 0.8 meters. The original Gaofen-2 satellite images are preprocessed, cropped, annotated in the range of 2000 ∗ 2000 pixels, and annotated various image types into ground truth images with different colors. According to the landform characteristics of Chenzhou, the species are divided into seven categories: cultivated land, road, forest land, buildings, water area, ridge and ditch, and others. The dataset contains 12,000 images, and the length and width of each image are 256 × 256. Randomly select 10,000 pictures as the training set and the remaining 2000 pictures as the test set.  Figure 9 shows the partial data cut into a uniform size from a large remote sensing image.

### 3.2. Preprocessing and Experiment Setup

In the deep learning network, it is easy to cause memory overflow when large remote sensing images to be classified are directly input into the network model. It is difficult for the model to identify the original data without preprocessing. Furthermore, training a deep learning network model needs lots of training data, however, labeling geographic information in satellite remote sensing images is a very complicated and time-consuming task, and labor costs are too high, making it difficult to produce large datasets. Additionally, for avoiding overfitting because of the small amount of data in the training data set in the process of deep learning neural network training, the existing training set needs to be enhanced and expanded. The image sizes of high-resolution remote sensing datasets are also inconsistent. Therefore, for a high-resolution remote sensing image, it needs to be cut into small images of uniform size as an experimental dataset. The pretreatment process is as follows:

1. Firstly, set the dataset image to the output image of the specified size as needed.
2. Secondly, perform random window sampling with a window size of 256 × 256 on the image, i.e., randomly generate sampling coordinates, and then obtain an image with a size of 256 × 256 under the coordinates.
3. Finally, data enhancement is performed on the segmented images, and image transformation operations are performed, such as rotation, vertical flipping, horizontal flipping, blurring, corrosion, random gamma transformation, bilinear filtering, and adding noise at random.

After the above data preprocessing and data expansion, the amount of data in the training set has become 6 times that of the original dataset, which reduces the risk of network overfitting in a way.

To ensure the reliability of the performance comparison of different network models, the experiments in this paper are carried out under the same development platform and hardware environment. The experimental equipment system is Windows 10, CPU (central processing unit) is Intel i7 3.30 GHz, GPU (graphics processing unit) is GeForce GTX 1080Ti (11G), GPU environment is CUDNN 10.0 and CUDA 10.0, the development platform is PyCharm, the programming language is Python, and the framework is Pytorch. The batch size of the test set is 4, and the batch size of the training set is also 4.

### 3.3. Evaluation Criteria

There are a variety of evaluation criteria used in semantic segmentation models. The evaluation criteria adopted in this paper are those adopted by most semantic segmentation models, including frequency weighted intersection (FWIU), pixel accuracy (PA), and mean intersection (MIOU) as performance indicators [4]. The evaluation criteria of frequency weighted intersection-over-union are defined as multiplying the frequency of each category as the weight with the intersection-over-union of each category and finally to sum. The evaluation criteria of pixel accuracy are defined as the ratio of correctly marked pixels to the total pixels. The evaluation criteria of mean intersection-over-union refer to the ratio of the intersection and union of the two sets of real and predicted values. Assume that the number of pixel categories is *K* + 1. The formulas of PA, MIOU, and FWIU are as follows:

(11) $$\begin{array}{c} PA=\frac{\sum_{i=0}^{k}P_{ii}}{\sum_{i=0}^{k}\sum_{j=0}^{k}P_{ij}},\\ MIOU=\frac{1}{k+1}\sum_{i=0}^{k}\frac{P_{ii}}{\sum_{j=0}^{k}P_{ij}+\sum_{j=0}^{k}P_{ji}-P_{ii}},\\ FWIU=\frac{1}{\sum_{i=0}^{k}\sum_{i=0}^{k}P_{ij}}\sum_{i=0}^{k}\frac{P_{ii}}{\sum_{j=0}^{k}P_{ij}+\sum_{j=0}^{k}P_{ji}-P_{ii}}. \end{array}$$

Among them, *P*_*ii*_ represents the number of class *i* pixels that are correctly classified, and *P*_*ij*_ represents the number of class *i* pixels classified as class *j*.

In addition, the precision, recall, and F1-score indicators in image classification are used in the experiment to evaluate the prediction effect of a single category. TP is defined as the model correctly predicted class *i*. TN is defined as the negative sample predicted correctly by the model. Defining FP as a negative sample is incorrectly predicted by the model to be a positive sample. Define FN as the class *i* is predicted to be other classes. Then, the precision is defined as follows:

(12) $$\begin{array}{c} \mathrm{Precision=}\frac{\mathrm{TP}}{\mathrm{TP+FP}}. \end{array}$$

Recall is defined as follows:

(13) $$\begin{array}{c} \mathrm{Recall=}\frac{\mathrm{TP}}{\mathrm{TP+FN}}. \end{array}$$

F1-score is defined as the harmonic mean of precision and recall, which is as follows:

(14) $$\begin{array}{c} F_{1}=\frac{1}{2}\left(\frac{1}{\mathrm{Precision+Recall}}\right). \end{array}$$

### 3.4. Experimental Results

In this paper, nine kinds of SCU-Nets are designed and tested on the dataset. The effect of depth and upsampling methods on the segmentation performance of SCU-Nets is studied. The experimental results are displayed in Table 1. The optimal experimental results are bolded.

According to the above table, the performance of SCU-Net using the C structure as the upsampling method is lower than the model using the other two structures. SCU-Net-102-A has the best comprehensive performance in the dataset. PA and MIOU are the highest, i.e., 91.53% and 55.84%, respectively. The MIOU of SCU-Net-102-A is the highest, which is 55.84%. It is 0.95% and 1.43% higher than SCU-Net-51-A and SCU-Net-153-A individually.

The results show that the depth of SCU-Net should be moderate, while scaling shallower or deeper may cause the performance of the network model to decrease. Meanwhile, SCU-Net-51-A is compared with other networks for studying the influence of parameters on network performance. Further comparisons are also conducted with the classic semantic segmentation neural networks DeepLab, U-Net, SegNet, FCN, Dilated, and the most recent networks FC-DenseNet and DFCN121. For the model obtained when the CFWE module in SCU-Net-102-A was deleted, a comparative experiment was carried out to verify the effectiveness of the CFWE module. The experimental comparison results are shown in Table 2. The optimal experimental results are bolded.

As can be seen from the above table, SCU-Net-102-A without a CFWE module is significantly lower than that of SCU-Net-102-A with CFWE module, and the parameters of the three CFWE modules are only 10,000. Hence, it can be inferred that the CFWE module has very few parameters and can greatly improve the performance of SCU-Net. DeepLabV3 uses and improves the ASPP module, which has a good effect on the GF-2 dataset, however, the performance is still lower than SCU-Net, and DeepLabV3 has many more model parameters than SCU-Net-102-A. FCN-8s achieved pixel classification by abandoning the fully connected layer of the traditional neural network and made great success on the GF-2 dataset with very few parameters. SegNet is a semantic segmentation network that improves VggNet-16 and is based on the FCN network. At the same time, it introduces the encoder-decoder structure, which has achieved good results on the GF-2 dataset, and the number of parameters is more than SCU-Net-51-A. U-Net was put forward to settle the matter of semantic segmentation of medical images. A U-shaped network structure was proposed to obtain location information and context information simultaneously. Although the parameters of U-Net are very few, it performs poorly on the GF-2 dataset. FC-DenseNet and DFCN121 introduced DenseNet into the model of semantic segmentation. At the same time, regardless of the number of other network parameters, SCU-Net performance is better than theirs. SCU-Net-51-A has low parameters and high performance. It shows that SCU-Net has better performance and lower model complexity and can be more targeted to complete the task of semantic segmentation of satellite remote sensing images.

To evaluate the application effect of the network in actual remote sensing images, use 2000 remote sensing images of 256 × 256 size as a test.  Table 3 lists the predicted pixels corresponding to 7 classes in the test images in detail. The optimal experimental results are bolded. Class 0–6 in the dataset, respectively, represent the background (cultivated land), forest land, others, water area, buildings, road, and furrow. The best experimental results are shown in bold. Meanwhile, the precision, recall, and F1-score of SCU-Net-102-A and DFCN121C models are compared. The precision and recall retain two decimal places, and the F1-score retains three decimal places.

It can be seen from Table 3 that all kinds of F1 scores predicted by the SCU-Net-102-A model are higher than those predicted by the DFCN121C model, except the “others” class. In addition, the forest F-score predicted by the SCU-Net-102-A model is the highest, which is 0.952. The corresponding forest land predicted precision reached 97.10%. At the same time, it can be found that the prediction effect of others in Table 3 is not so ideal mainly because of the combination of classes during manual labeling. There are not many experimental data samples of bare land or wasteland, and the geographical characteristics are not very obvious. Hence, the prediction results will be affected to some extent.

### 3.5. Experiments Analysis

The experimental results show that the PA and MIOU of SCU-Net-102-A are the highest, which are 91.53% and 55.84%, respectively. After comprehensive consideration, SCU-Net-102-A is chosen to compare with other typical semantic segmentation networks and the more recent semantic segmentation networks. It is found that the comprehensive performance of the network is better than other networks. Judging from the experimental results, the network depth should be kept appropriate in the task of semantic segmentation of satellite remote sensing images. Too few network layers make it difficult to extract sufficient features, and too many network layers will cause vanishing gradient problem or gradient explosion problem. The problems of gradient dispersion and gradient explosion can be solved to some extent by batch normalization, and the degradation problem can be alleviated by jumping connection. The CDeConv upsampling module uses a point convolutional layer, which improves the feature extraction capability of the network on the basis of reducing the number of network parameters. In addition, the attention mechanism module CFWE module, which uses skip connections to settle the matter of network degradation to some extent, is introduced. Simultaneously, the CFWE module learns the channel weight coefficients using the attention mechanism, which enhance the feature extraction capability of the network and achieves a better image segmentation effect. SCU-Net-102-A and DFCN121C networks are selected for experiments to compare and predict the effects of different categories. The precision of the SCU-Net-102-A model for forest land prediction is 97.10%, and the recall is 93.42%. The corresponding F1-scores reached 0.952, which is the best among the 7 classes, and these three values are higher than those of the DFCN121C model. At the same time, all kinds of F1 scores predicted by SCU-Net-102-A are higher than those predicted by DFCN121C, except for the “others” class. Combined with the experimental results, it can be proved that SCU-Net-102-A is better than DFCN121C in predicting each.

### 3.6. Visualization of Segmentation Results

The visualization diagram of the SCU-Net-A test output is shown in Figure 10. The first row is the input image of the test set, the second row is the ground truth, the third row is the image predicted by DFCN121C, and the fourth row is the image predicted by SCU-Net-102-A. In the experiment, two remote sensing images with a size of 1856 × 1856 were selected, and the SCU-Net-102-A and DFCN121C network models were used for prediction. The red rectangle indicates the prediction error, the yellow rectangle indicates the prediction effect on the water category, and the rose-red rectangle indicates the prediction effect on the road category.

On the whole, the prediction effect of SCU-Net-102-A is better than the image predicted by DFCN121C. In the first raw image, the waters are marked as bare ground because of human labeling errors. Both SCU-Net-A and DFCN121C can correctly predict waters, however, it is clear that SCU-Net-102-A understands the details better, as shown by the yellow boxes in the first column of Figure 10. As can be seen from the above figure, both SCU-Net-102-A and DFCN121C can predict unlabeled waters, however, the boundary information of SCU-Net-102-A is better than that of DFCN121C. It is indicated by the yellow box in the second column of Figure 10. Furthermore, it is experimentally found that DFCN121C predicts more misinformation than SCU-Net-102-A, as shown by the red boxes in Figure 10. In addition, there are unmarked roads in the original image in the second column, however, both SCU-Net-102-A and DFCN121C have learned this road information, and it can be seen from the figure that SCU-Net-102-A is better than DFCN121C as it learned more about the road category, as shown by the rose-red box in Figure 10. It shows that SCU-Net-102-A has a strong generalization ability in the semantic segmentation of high-resolution remote sensing images.

## 4. Conclusions

This paper proposes a new semantic segmentation model for high-resolution remote sensing images based on CNNs. A new upsampling module CDeConv is proposed in this network model, and the attention module CFWE is used to improve the feature extraction ability of the network. In the experiment of this paper, the GF-2 satellite remote sensing image of Chenzhou in 2016 is used, and the ground truth was labeled manually. Finally, there were 7 categories of classified objects in the dataset. By analyzing the experimental results, it is concluded that SCU-Net-102-A has the highest value, and its PA and MIOU are 91.66% and 55.61%, respectively. The precision of SCU-Net-102-A for woodland prediction is 97.10%, and the corresponding F1-score is 0.952, which is the highest F1-score among the seven categories. It can achieve accurate segmentation of complex targets in GF-2 image classification tasks. The model designed in this paper is designed to detect the changes in forest land and water area in Chenzhou, China, and to provide help for the protection and development of forest and water environment. It is hoped that more satellite remote sensing images of the same kind can be obtained in the future, and higher-quality segmentation datasets can be generated to further train SCU-Net to improve its versatility and segmentation performance.

## Figures and Tables

**Figure 1:** The structure of FCN.

**Figure 2:** The structure of CFWE.

**Figure 3:** The structure of CDeConv.

**Figure 4:** The structure of SCU-Net.

**Figure 5:** Remote sensing image segmentation flowchart (the convolutional layer is represented by blue blocks, the pooling layer is represented by green blocks, the superimposed convolutional layer is represented by orange blocks, the yellow block represents the CFWE, and the gray block represents the upsampling operation).

**Figure 6:** Comparison of SCU-net's parameters.

**Figure 7:** Comparison of floating-point operations (FLOPs).

**Figure 8:** High-resolution remote sensing image.

**Figure 9:** Cases of satellite remote sensing images (the spatial resolution is 0.8 meters).

**Figure 10:** Prediction maps of the SCU-net-102-A and DFCN121C (the ground truth map is divided into 7 classes: 0 for background, 1 for woodland, 2 for bare land or wasteland, 3 for waters, 4 for buildings, 5 for roads, and 6 for furrows. The first row is the original high-resolution remote sensing image, the second row is the ground truth, the third row is the DFCN121C prediction map, and the fourth row is the SCU-net-102-A prediction map).

**Table 1:** The performance of different depth SCU-nets.

Model	PA (%)	MIOU (%)	FWIU (%)
SCU-net-51-A	91.30	54.99	**85.95**
SCU-net-102-A	**91.53**	**55.84**	85.83
SCU-net-153-A	91.58	54.51	85.98
SCU-net-51- B	91.16	54.56	85.62
SCU-net-102- B	91.43	54.76	85.69
SCU-net-153-B	91.10	54.54	85.16
SCU-net-51-C	91.25	53.74	85.49
SCU-net-102-C	91.06	54.37	85.29
SCU-net-153-C	91.15	54.24	85.45

**Table 2:** Performance of different depth SCU-nets.

Model	PA (%)	MIOU (%)	FWIU (%)	PRM (m)
SCU-net-102-A	**91.53**	**55.84**	85.83	42.71
NoSCU-net-102-A	91.36	53.77	85.52	42.70
DeepLabV3 [20]	87.87	49.70	81.80	58.00
FCN-8s [10]	90.55	51.16	84.61	14.70
SegNet [17]	91.17	50.60	85.35	28.40
U-net [16]	89.65	44.50	83.55	13.40
FC-DenseNet [11]	84.99	51.67	**90.85**	**9.40**
DFCN121 [13]	91.28	54.03	85.69	17.00
SCU-net-51-A	91.30	54.99	85.95	23.72

**Table 3:** Labeling results of SCU-net-102-A and DFCN121C for each class on the GF-2 dataset.

Model		Cultivated land	Forest land	Others	Water area	Building	Road
Predict pixels		22288550	92223235	199063	11547582	2982585	1830985

Predict pixels (TP)	SCU-net-102-A	15161346	89547666	113169	11183917	886270	1517840
	DFCN121C	14883805	89361908	117344	11255276	1999480	289870

Predict pixels (FP)	SCU-net-102-A	7127204	2675569	85894	363665	2096315	313145
	DFCN121C	7404745	2861327	81719	292306	983105	1541115

Precision	SCU-net-102-A	68.02%	**97.10%**	43.15%	96.85%	70.29%	82.90%
	DFCN121C	66.78%	96.90%	58.95%	97.47%	67.04%	84.17%

Recall	SCU-net-102-A	82.88%	93.41%	50.98%	92.15%	86.90%	72.87%
	DFCN121C	83.20%	93.16%	50.11%	90.71%	86.89%	70.87%

F1-score	SCU-net-102-A	0.747	**0.952**	0.467	0.944	0.777	0.776
	DFCN121C	0.741	0.949	0.541	0.939	0.757	0.769

## Data Availability

The dataset can be obtained from the corresponding author upon request.

## References

[1] Yao C., Luo X., Zhao Y., Wei Z., Chen X. A review on image classification of remote sensing using deep learning.

[2] Liu Y., Piramanayagam S., Monteiro S. T., Saber E. (2019). Semantic segmentation of multisensor remote sensing imagery with deep ConvNets and higher-order conditional random fields. *Journal of Applied Remote Sensing*.

[3] Baranoski G., Kimmel B. W., Varsa P. (2019). Assessing the impact of porosity variations on the reflectance and transmittance of natural sands. *Journal of Applied Remote Sensing*.

[4] Krizhevsky A., Sutskever I., Hinton G. ImageNet classification with deep convolutional neural networks.

[5] Wang W., Yang Y., Wang X., Wang W. Z., Li J. (2019). Development of convolutional neural network and its application in image classification: a survey. *Optical Engineering*.

[6] Wang W., Li Y., Zou T., Wang X., Luo Y. (2020). A novel image classification approach via dense-mobilenet models. *Mobile Information Systems*.

[7] Wang W., Liu H., Li J., Nie H., Wang X. (2020). Using CFW-net deep learning models for X-ray images to detect COVID-19 patients. *International Journal of Computational Intelligence Systems*.

[8] Xue Y., Wang Y., Liang J., Slowik A. (2021). A self-adaptive mutation neural architecture search algorithm based on blocks. *IEEE Computational Intelligence Magazine*.

[9] Xue Y., Jiang P., Neri F., Liang J. (2021). A multi-objective evolutionary approach based on graph-in-graph for neural architecture search of convolutional neural networks. *International Journal of Neural Systems*.

[10] Long J., Shelhamer E., Darrell T. (2015). Fully convolutional networks for semantic segmentation. *IEEE Transactions on Pattern Analysis and Machine Intelligence*.

[11] Ren S., He K., Girshick R., Sun J. (2017). Faster R-CNN: towards real-time object detection with region proposal networks. *IEEE Transactions on Pattern Analysis and Machine Intelligence*.

[12] Wang W., Tang C., Wang X., Luo Y., Hu Y., Li J. (2019). Image object recognition via deep feature-based adaptive joint sparse representation. *Computational Intelligence and Neuroscience*.

[13] Lécun Y., Bottou L., Bengio Y., Haffner P. (1998). Gradient-based learning applied to document recognition. *Proceedings of the IEEE*.

[14] Simonyan K., Zisserman A. (2014). Very deep convolutional net-works for large-scale image recognition.

[15] Szegedy C., Liu W., Jia Y. Going deeper with convolutions.

[16] He K., Zhang X., Ren S. Deep residual learning for image recognition.

[17] Simon J., Drozdzal M., Vazquez D., Romero A., Bengio Y. The one hundred layers tiramisu: fully convolutional DenseNets for semantic segmentation.

[18] Huang G., Liu Z., Maaten L. V. D., Weinberger K. Q. Densely connected convolutional networks.

[19] Wang W., Yang Y. J., Li J., Hu Y., Wang W. (2020). Woodland Labeling in Chenzhou, China via deep learning approach. *International Journal of Computational Intelligence Systems*.

[20] Hamida A., Benoît A., Lambert P., Klein L. Deep learning for semantic segmentation of remote sensing images with rich spectral content.

[21] Wang W., Jiang Y., Luo Y., Li J., Zhang T. (2019). An advanced deep residual dense network (DRDN) approach for image super-resolution. *International Journal of Computational Intelligence Systems*.

[22] Ronneberger O., Fischer P., Brox T. U-Net: convolutional networks for biomedical image segmentation.

[23] Badrinarayanan V., Kendall A., Cipolla R. (2017). SegNet: a deep convolutional encoder-decoder architecture for image segmentation. *IEEE Transactions on Pattern Analysis and Machine Intelligence*.

[24] Chen L. C., Papandreou G., Kokkinos I., Murphy K., Yuille A. L. (2014). Semantic image segmentation with deep convolutional nets and fully connected CRFs. *Computer Science*.

[25] Chen L.-C., Papandreou G., Kokkinos I., Murphy K., Yuille A. L. (2018). DeepLab: semantic image segmentation with deep convolutional nets, Atrous convolution, and fully connected CRFs. *IEEE Transactions on Pattern Analysis and Machine Intelligence*.

[26] Chen L. C., Papandreou G., Schroff F., Adam H. (2017). Rethinking atrous convolution for semantic image segmentation.

[27] Chen L.-C., Zhu Y., Papandreou G., Schroff F., Adam H. Encoder-decoder with atrous separable convolution for semantic image Segmentation.

[28] Chollet F. Xception: deep learning with depthwise separable convolutions.

[29] Mitra P., Uma Shankar B., Pal S. K. (2004). Segmentation of multispectral remote sensing images using active support vector machines. *Pattern Recognition Letters*.

[30] Bilgin G., Erturk S., Yildirim T. (2011). Segmentation of hyperspectral images via subtractive clustering and cluster validation using one-class support vector machines. *IEEE Transactions on Geoscience and Remote Sensing*.

